RETRACTED

# Efficient Approach towards Detection and Identification of Copy Move and Image Splicing Forgeries Using Mask R-CNN with MobileNet V1

**DOI:** 10.1155/2022/6845326

**Published:** 2022-01-05

**Authors:** Kalyani Dhananjay Kadam, Swati Ahirrao, Ketan Kotecha

**Affiliations:** ^1^Symbiosis Institute of Technology, Symbiosis International (Deemed University), Pune, Maharashtra 412115, India; ^2^Symbiosis Centre for Applied Artificial Intelligence, Symbiosis International (Deemed University), Pune, Maharashtra 412115, India

## Abstract

With the technological advancements of the modern era, the easy availability of image editing tools has dramatically minimized the costs, expense, and expertise needed to exploit and perpetuate persuasive visual tampering. With the aid of reputable online platforms such as Facebook, Twitter, and Instagram, manipulated images are distributed worldwide. Users of online platforms may be unaware of the existence and spread of forged images. Such images have a significant impact on society and have the potential to mislead decision-making processes in areas like health care, sports, crime investigation, and so on. In addition, altered images can be used to propagate misleading information which interferes with democratic processes (e.g., elections and government legislation) and crisis situations (e.g., pandemics and natural disasters). Therefore, there is a pressing need for effective methods for the detection and identification of forgeries. Various techniques are currently employed for the identification and detection of these forgeries. Traditional techniques depend on handcrafted or shallow-learning features. In traditional techniques, selecting features from images can be a challenging task, as the researcher has to decide which features are important and which are not. Also, if the number of features to be extracted is quite large, feature extraction using these techniques can become time-consuming and tedious. Deep learning networks have recently shown remarkable performance in extracting complicated statistical characteristics from large input size data, and these techniques efficiently learn underlying hierarchical representations. However, the deep learning networks for handling these forgeries are expensive in terms of the high number of parameters, storage, and computational cost. This research work presents Mask R-CNN with MobileNet, a lightweight model, to detect and identify copy move and image splicing forgeries. We have performed a comparative analysis of the proposed work with ResNet-101 on seven different standard datasets. Our lightweight model outperforms on COVERAGE and MICCF2000 datasets for copy move and on COLUMBIA dataset for image splicing. This research work also provides a forged percentage score for a region in an image.

RETRACTED

## 1. Introduction

Digital images are used in almost every domain, such as public health services, political blogs, social media platforms, judicial inquiries, education systems, armed forces, businesses, and so on. Rapid advances in digital technology have led to the creation and circulation of a vast amount of images over the last few years. With the use of image/photo editing tools like Canva, CorelDRAW, PicMonkey, PaintShop Pro, and many other applications, it has become very easy to manipulate images and videos. Such digitally altered images are a primary source for spreading misleading information, impacting individuals and society. The deliberate manipulation of reality through visual communication with the aim of causing harm, stress, and disruption is a significant risk to society, given the increasing pace at which information is shared through social media platforms such as Twitter, Quora, and Facebook. It becomes a significant challenge for such social media platforms to identify the authenticity of these images. For example, cybersecurity experts [1] have reported that hackers have the ability to access patient's 3-D medical scans and can edit or delete images of cancerous cells. In a recent study, surgeons were misled by scans modified with AI software, possibly leading to a high risk of misdiagnosis and insurance fraud. In addition, manipulated images related to politics [2] distributed across social media platforms have the potential to mislead and influence public perceptions and decisions. For example, studies have shown that that particular types of images are likely to be reused and, in certain cases, exploited in online terrorism communication channels through media sources [3–5]. Image alteration becomes too easy using image editing software and even altering the original image in such a way that forensic investigators will not be able to identify the changes in the image. The major camera manufacturers use digital certificates to solve this issue. However, some companies have generated forged images taken from Canon and Nikon camera models. These fake images are passed through manufacturer verification software to perform their authenticity test [6].

Therefore, there is a need to develop a forgery detection technique that detects and identifies forgeries to resolve these challenges. Many forgery detection techniques shown in Figure 1 have been developed to authorize a digital image. These techniques are usually split into two types, referred to as active and passive detection techniques [7–9]. In active detection, a message digest or digital signature [10–14] is injected inside an image when it is created. In this forgery detection technique, statistical information such as mean, median, and mode is inserted into an image using some encryption method; this information is then retrieved from the image at the receiving side using a decryption method to check its authenticity [15]. In passive detection, changes in the entire image and local features are identified. It does not leave any visual clues of forgery, but it alters the statistical information of an image. It verifies the structure and content of an image to determine its validity.

RETRACTED

Passive detection is classified into forgery type-dependent and independent detection techniques. Forgery-dependent techniques are popular as they handle particular kinds of image forgeries, like image splicing and copy move. Copy move [16] duplicates a part of an image in several positions within the same image. Image splicing is the process of merging two or multiple images to produce a new image [17]. There are many research studies into the identification of copy move and image splicing forgeries. The traditional forgery detection techniques specified in the literature of image forgery detection depend on the image's frequency domain properties or statistical information. These techniques utilize relevant features, and then these features are used to differentiate the original image from the forged image. These techniques mainly focus on designing complex handcrafted features. However, it is difficult to identify which feature should be extracted for detecting forgery.

Some research works have used various machine learning algorithms for forgery detection. Conventional machine learning (ML) algorithms like logistic regression, SVM, and *K*-means clustering consider every pixel of the image as an individual dimension, thereby formulating image classification as a geometry problem [18]. Images are converted into high-dimensional vectors, and classification boundaries are learned through these algorithms. Unfortunately, such algorithms are often unable to learn very complex boundaries, leading to poor performance in image classification. Few machine learning algorithms that use distance metrics, such as *K*-nearest neighbours and *K*-means clustering [19], are computationally expensive because they require large dimensional vector spaces.

Rapid developments in computational capabilities such as processing power, memory space, and power consumption have enhanced the efficiency and cost-effectiveness of computer vision-based applications. DL helps computer vision researchers to gain better accuracy in image classification [20], semantic segmentation [21], and object identification [22] compared to conventional CV techniques. DL algorithms are more versatile as compared to traditional computer vision algorithms, which are more domain-specific. For specific applications, pretrained CNN models are used where the weights are already learned over large datasets (which contain millions of images). These models are open-sourced for all developers, and only the last few layers need to be modified in order to fine-tune for a specific application [23, 24]. Various DL networks have been proposed in the computer vision area, including AlexNet [25]; in 2012, it won the *ImageNet Large Scale Visual Recognition Challenge*, thereby increasing classification accuracy by 10% over traditional machine learning algorithms. *VGGNet* [26] was proposed by the University of Oxford's Visual Geometry Group in 2014, and *GoogLeNet* [27] and *ResNet* [28] were proposed in 2015. Several DL networks in computer vision discussed above are becoming increasingly complex to achieve greater accuracy. The aforementioned DL network's parameters increase exponentially, making these networks more reliant on computationally efficient graphical processing units (GPUs) [29]. To address the challenges of existing work, this work contributes a lightweight deep learning classification network based on *MobileNet V*1 [30]. This network is built on the depthwise separable convolution principle [31, 32], which minimizes network parameters and computational complexity in the convolution processing operation, resulting in a lightweight network.

RETRACTED

The significant contributions of this research work are as follows:

- Development of DL architecture for detection and identification of copy move and image splicing forgeries.
- Detection and identification of copy move and image splicing forgeries using Mask R-CNN with MobileNet V1, a lightweight network and computationally less expensive.
- Evaluation of Mask R-CNN with MobileNet V1 on seven different datasets such as COVERAGE [33], CASIA 1.0 [34], CASIA 2.0 [34], COLUMBIA [35], MICC F220 [36], MICC F600 [36], and MICC F2000 [36].
- Comparative analysis of the proposed work with ResNet-101 on different standard datasets.
- Estimation of the percentage score for a region of a forged image using Mask R-CNN and MobileNet V1.

This paper is structured as follows.  Section 1 presents an introduction, related work is outlined in Section 2, Section 3 shows the proposed architecture, the details of the datasets are outlined in Section 4, dataset annotation is given in Section 5, Section 6 outlines implementation details, Section 7 shows the results, and Section 8 presents the conclusion.

RETRACTED

## 2. Related Work

This section specifies related work for copy move using DL, image splicing using DL, and DL networks for computer vision.

### 2.1. Copy Move

The research work in [37] uses CNN for detecting copy move and image splicing forgeries. For extracting features from patches, the CNN network had been pretrained on labeled images. The SVM model is then trained using the extricated features. The research work in [38] uses CNN along with a deconvolutional network for copy move forgery detection. The test image is divided into blocks, and then CNN is used to extract the features from these image blocks. Self-correlations between these blocks are then calculated. After that, the matched points between blocks are localized, and finally, the deconvolutional network reconstructs the forgery mask. This copy move forgery detection (CMFD) technique is more robust against postprocessing operations such as affine transformation, JPEG compression, and blurring.

The study in [39] uses Mask R-CNN and the Sobel filter for detection and localization of copy move and image splicing forgeries. Here the employed Sobel filter allows predicted masks to identify gradients that are close to those of the real mask.

The work in [40] uses six convolutional layers and three FC layers. Here batch normalization is used in all the convolution layers and dropout in the FC layers (except in the last layer). CoMoFoD and BOSSBase datasets are used for evaluation of this technique which achieves an accuracy of 95.97% and 94.26%, respectively, on these datasets. The research study in [41] uses various processes such as segmentation, feature extraction, and dense depth reconstruction, finally identifying the tampered area for copy move forgery detection. Here forged image is segmented with simple linear iterative clustering (SLIC). Then, from these segmented patches, features from various scales are extracted using VGG-16. These features are used to reconstruct the dense depth of the image pixel which aids in the matching of the forged and original region. After the reconstruction process, the ADM (adaptive patch matching) technique is applied to find out the matched regions. The majority of the suspicious regions are apparent at the end of this operation. During this process, the unforged regions are removed and the forged regions are visible. The MICC F220 dataset was used in the experiments, which achieves a precision of 98%, recall of 89.5%, *F*_1_-score of 92%, and accuracy of 95%. The main contribution of the research in [42] is the development of a CNN for categorizing images into two groups: authentic and forged. Image features are extracted and feature maps are created by the CNN. The CNN takes the average of the produced feature maps and searches for feature correspondences and dependencies. The trained CNN is then used to classify the images. This technique has been tested on MICC F220, MICC F2000, and MICC F600 datasets in a variety of copy move situations, including single and multiple cloning with varying cloning regions, and achieved 100% accuracy and zero log loss using 50 epochs. The earlier research work shows remarkable performance but suffers from a few challenges such as generalization issues due to significant reliance on training data and the necessity for suitable hyperparameter selection. To address this issue, the researchers proposed [43] two deep learning techniques: a custom design of architecture and a transfer learning model for copy move forgery detection. To address the challenge of generalization, different standard datasets were employed. In the custom design technique, five architectures were designed with different depths (architectures with convolution layers up to five with two FC layers were used). The second technique is transfer learning for which the VGG-16 pretrained model is used. The pretrained model (pretrained with VGG-16) differs from custom design model in terms of depth, the number of filters in the convolutional layers, the activation function, and the number of convolutional layers before the pooling layer. The VGG-16 model by transfer learning obtained metrics is around 10% higher than the model by custom design, but it required more inference time.

RETRACTED

The research study in [44] uses MobileNet V2 for the detection of copy move forgery with postprocessing operations related to visual appearance and geometrical operations. The MobileNet V2 model is a notable performer with TPR and FPR of 84% and 14.35%, respectively. Experiments show that the improved MobileNet V2 CNN framework is robust and resource-friendly. The work in [45] uses a DL technique based on a hybrid ConvLSTM and CNN. The main goal of this study was to develop and improve a deep learning classification model for distinguishing between authentic and forged digital image forgeries. This method extracts image features by a sequence number of convolution (CNV) layers, ConvLSTM layers, and pooling layers, matching features and detecting copy move forgery. This technique is then tested on MICC F220, MICC F2000, MICC F600, and SATs-130. To address the generalization issue, a new dataset was created by merging the aforementioned datasets. The model developed in this research work offers good performance with low computing costs.

In [46], the researchers presented a framework for classifying input images as authentic or forged by combining the image transformation techniques along with pretrained CNN. The three image transformation techniques such as LBP (local binary pattern), DWT (discrete wavelet transform), and ELA (error level analysis) were used to extract appropriate features. In this framework, ELA is used to transform images and then these images are used to train a CNN to detect forged images. The model's training potential is further enhanced by using transfer learning to initialize the weights of the CNN with pretrained VGG-16. The experiments are performed on public benchmark datasets. The model was tested on generalized images. The research work in [47] uses the CNN model which is developed using multi-scale input with multiple stages of convolutional layers. These layers are divided into two blocks, i.e., encoder and decoder. The encoder block combines and downsamples derived feature maps from many levels of convolutional layers. Similarly, extracted feature maps in decoder blocks are concatenated and upsampled. The final feature map is employed to distinguish pixels as forged or non-forged using a sigmoid activation function. Two publicly available datasets are utilized to validate the model.

RETRACTED

### 2.2. Image Splicing

The study in [48] uses the FCN model for detecting image splicing in an image. The single-task FCN is trained with a surface label that classifies an image's pixel as spliced or authentic. But single-task FCN generates coarse localization output for some cases. The improved edge MFCN performs better than SFCN and MFCN. It is trained with surface labels and boundary labels, and it uses a surface label and edge probability map to localize the spliced field. The study in [49] employed the conditional generative adversarial network (cGAN) to detect spliced forgeries in satellite images. It had a high degree of accuracy in detecting and locating spliced objects.

The research work in [50] is based on a local feature descriptor learned by a deep convolutional neural network (CNN). A two-branch CNN is used to automatically train hierarchical representations from RGB color or grayscale test images using the local descriptor. The proposed CNN model's first layer is used to suppress image content effects and extract the various and expressive residual features, which is specifically considered for image splicing detection. The first layer's kernels are initialized with an improved initialization method based on the SRM. The proposed CNN model's generalization ability is improved by combining the contrastive loss with cross-entropy loss. In order to acquire the final discriminative features of the test image for image splicing detection with SVM, an effective feature fusion approach known as block pooling was used with the blockwise dense features which were retrieved by the pretrained CNN-based local descriptor on a test image. For image splicing, localization of spliced region is further developed based on the pretrained CNN model by including the fully connected conditional random field (CRF). Extensive testing on many public datasets reveals that the proposed CNN-based strategy outperforms the state-of-the-art algorithms not only for image splicing detection and localization performance but also in JPEG compression robustness.

RETRACTED

In [51], the researchers offer a new image splicing detection system that uses ResNet-Conv, a new deep learning backbone architecture. ResNet-Conv is created by substituting a set of convolutional layers for the feature pyramid network in ResNet-FPN. The initial feature map is generated using this new backbone, which is then used to train the Mask-RCNN to build masks for spliced regions in forged images. ResNet-50 and ResNet-101 are two distinct ResNet architectures that are considered. Several postprocessing operations were employed on the input images to get more realistic forged images. Using a computer-generated image splicing dataset, the proposed network is trained and tested, and it is found to be more efficient than alternative networks. The DL-based image splicing technique proposed in [52] used a convolutional neural network and a weight combination mechanism. In this technique, YCbCr features, edge features, and PRNU features were merged, and their weight settings were automatically changed during the CNN training process until the best ratio was achieved.

The research work in [53] uses ResNet-50 pretrained deep learning network and a quantum variational circuit. Using Xanadu's PennyLane quantum simulator and the PyTorch DL framework, researchers presented a comparative empirical analysis of classical versus quantum transfer learning approaches. The model was tested on IBM's genuine quantum processor, the ibmqx2. The quantum processor (accuracy = 85% and recall = 87.18%) and simulator (accuracy = 81.94% and recall = 91.67%) outperformed conventional computers (accuracy = 80.57% and recall = 89.11%).

In [54], two techniques are used for image splicing detection. Firstly, the “Noiseprint” technique is used which suppresses the image content and exposes the tampering artifacts in the spliced images more accurately. Secondly, the ResNet-50 network is used as a feature extractor which learns the distinguishing features between the authentic and spliced images. Finally, the SVM classifier is used to classify the images as spliced or authentic. The future work of this research focuses to distinguish authentic videos (videos recorded using a single camera) from spliced videos (videos created by merging different videos). It also locates the exact spliced region in a spliced region. The research study in [55] introduces a convolution neural net-based technique for the selection of features, which eliminates the time-consuming job of manually selecting image features. The feature vector is then loaded into a dense classifier network to assess if an image is authentic or spliced. The proposed model is trained, validated, and tested on CASIA v2.0. The experimental results show that the proposed technique outperforms the current state-of-the-art techniques. The limitation of this technique is that it is not able to locate spliced region.

RETRACTED

The research study in [56] uses color illumination, deep convolution neural networks, and semantic segmentation to detect and localize image splicing forgery. After the preprocessing step, color illumination is employed to apply the color map. The deep convolution neural network is used to train VGG-16 with two classes using the transfer learning approach. This research study determined whether a pixel is authentic or forged one. In order to locate forged pixels, semantic segmentation was used which is trained on images using color pixel labels. The technique used in [57] integrates handcrafted features based on color characteristics and deep features using the image's luminance channel to get patterns for forgery detection. The quaternion discrete cosine transform of the image is used to compute 648-D Markov-based features in the first stream. The image's local binary pattern is extracted in the second stream using the YCbCr colorspace's luminance channel. Local binary feature maps are also input into the pretrained ResNet-18 model to get a 512-D feature vector named “ResFeats” from the model's convolutional base portion's last layer. An 1160-D feature vector is formed by combining the handcrafted features from stream I and ResFeats from stream II. A shallow neural network is used to perform classification. This technique was evaluated on the CASIA v1 and CASIA v2 datasets, and on these datasets, this fusion-based technique achieves 99.3% accuracy.

### 2.3. Deep Learning Networks for Computer Vision

In the field of computer vision, image segmentation is a famous topic for researchers. This process divides an image into different regions, and based on the characteristics of pixels of these regions, it specifies various objects of the image and its boundary. R-CNN [58], Fast R-CNN [59], Faster R-CNN [60], and Mask R-CNN [61] are variants of region-based CNN algorithms; these algorithms provide better segmentation in a reasonable amount of time. R-CNN algorithm [58] stood out among various algorithms when applied to VOC2007 data. R-CNN is utilized for object identification and classification in images, with bounding boxes for different image objects. In R-CNN [58], nearly two thousand region proposals are generated using a selective search algorithm, and they are wrapped to a fixed size. These wrapped proposals are then fed to CNN, which acts as an image feature extractor, extracting a predetermined-size image feature vector from each region. R-CNN extracts 4096-dimensional feature vector from each region proposal. The extracted features are then fed to SVM, which helps in classifying the presence of objects in the region. The bounding box's coordinates are estimated using a regressor.

RETRACTED

*Fast R-CNN* [59] is an object classification method, and detection method based on deep ConvNets uses two thousand ConvNets for each image region. A single deep ConvNet significantly speeds up feature extraction. Then, the softmax function is used for classification, which marginally outperforms *SVM*. *Faster R-CNN* [60] uses three networks for object detection. CNN is the first network that produces feature maps for the given input image. *An RPN* is a second network that generates a collection of bounding boxes called ROIs with more chances of having objects inside them. A final network takes feature maps from the convolutional layer and generates an object's bounding boxes as well as predicts its class. *Faster R-CNN* is improved by *Mask R-CNN* [61], which provides a mask for the individual region of interest.

Recent literature shows that there has been growing interest in developing small networks [62, 63]. Small networks are created using compression. There are two techniques for performing compression: (i) by tuning the network parameters to train the models and (ii) developing and training small size models. For the first method, various squeezing techniques like product *quantization* [63], *Huffman coding* [64], *pruning*, *vector quantization*, and *hashing* [65] have been suggested for reducing the size of the network. Pretrained networks could be shrunk, factorized, and compressed to get smaller networks. Distillation [66] is another compression model used to train small networks from larger networks. The second technique has gained popularity with the development of lightweight networks like *SqueezeNet* [67], *ShuffleNet* [68], and MobileNet V1 [30]. *SqueezeNet* [67] is a technique for building a tiny size network that significantly decreases network specifications and processing overhead by maintaining network efficiency*. ShuffleNet* [68] uses channel shuffling and point-group convolution to minimize network computation. *MobileNet V*1 [30] is based on the concept of depthwise separable convolution [30, 31]. Each channel's features are convolved separately, and then all features of different channels are spliced using 1 × 1 convolution. These lightweight networks minimize the total number of network parameters and computing costs. The following gaps are identified in the current literature on copy move and image splicing forgeries:

1. Detection and identification of passive forgeries such as copy move and splicing are computationally expensive due to the large number of parameters, storage, and computational cost.
2. Identification of percentage score for the image being forged.

RETRACTED

## 3. Proposed Architecture

This section shows the proposed architecture for detection and identification of copy move and image splicing forgeries and provides the forged percentage of a forged image. The proposed architecture has facilities for detection and identification of image forgeries such as copy move and image splicing and calculation of the forged percentage of given input image.

(i) *Detection and Identification of Image Forgeries like Copy Move and Image Splicing*. The approach involves the use of *Mask R-CNN* with *MobileNet V*1 [30].  Figure 2 depicts the architecture of the proposed system. In the first step, the proposed system takes an image as an input and performs feature extraction. RPN then provides the regions or image characteristics maps that may contain various objects. The image characteristics maps or regions come in various sizes, and ROI is used to convert them to a defined form. The second step is the detection step which specifies the class of forged object(s), such as copied or spliced, and it also creates bounding boxes around the forged object. The last step is segmentation which generates a mask around the forged object. Thus, the proposed model's output for the given input image is detection and identification of the forged object(s) with a bounding box and a classification of the type of forgery.
(ii) *Calculating the Forged Percentage of a Given Input Image*. The image forgery detection architecture is also used to calculate the forged percentage for a given image. The general formula for calculating a region's forged percentage is shown below.
  (1) $$\begin{array}{c} A=\text{number of pixels of the entire image,}\\ B=\text{number of pixels of the forged region,}\\ \text{forged percentage of region }=\frac{\left[A-B\right]}{\text{dimension of image}}\times 100. \end{array}$$
In the architecture, the forged regions are classified and localized using a bounding box and semantic segmentation that classifies each pixel. Every region of interest gets a polygon segmentation mask. By utilizing the predicted segmentation masks, the percentage of the individual mask area of the forged regions is calculated. The masks generated by the architecture are regarded as a binary image, so the forged region will be white (true), and the background will be black (false). To calculate the percentage of the area of the segmentation masks, firstly the number of pixels occupied by the forged region is calculated. This can be determined by counting the number of pixels belonging to a white color or by counting the number of pixels belonging to black color (background pixels) and subtracting it from the total number of pixels in the image. The total pixel count can be calculated by multiplying the width and height of the image. The final percentage of area is calculated by using the following equation:
  (2) $$\begin{array}{c} \%=\frac{\text{white pixel count}}{\text{total pixel count}}\;\times \;100. \end{array}$$
In case of an input image having multiple forged regions, the architecture will generate multiple polygon masks. So, for an image having three forged objects, three masks will be generated. To get the total percentage of the area of these three segmentation masks, first, the white pixel count of each individual mask is calculated.
  (3) $$\begin{array}{c} \text{Total white pixel count }=\sum_{i=1}^{n}\text{white pixel count of }{\text{mask}}_{i},\\ n=\text{number of masks.} \end{array}$$
Then, the final percentage can be calculated.
  (4) $$\begin{array}{c} \%\;=\;\frac{\text{total white pixel count}}{\text{total pixel count}}\;\times \;100. \end{array}$$
The architecture of the proposed system for detection, localization of copy move and image splicing forgery, and calculation of the forged percentage is explained below.

RETRACTED

### 3.1. MobileNet V1 [30]

In CV, CNN has become very common in the image classification and segmentation process. However, modern CNNs are becoming deeper and increasingly complex to achieve a greater degree of accuracy. MobileNet V1 reduces the size (in terms of the number of parameters) and complexity (in terms of multiplications and additions (multi-adds)) of the network. MobileNets are based on DSCLs, where each DSCL consists of two convolution types: depthwise convolution and pointwise convolution.  Figure 3 shows the standard convolution operation [32]. Each pixel of an image is multiplied by the number of filter channels and takes a total of the input pixels handled by the filter that slides through all the image's input channels. Depthwise separable convolution is shown in Figure 4. Image characteristics are learned only using input channels, and thus the output layer has an equal number of channels as the input channels. In depthwise separable convolution, kernels are split into smaller ones which yield the same result with fewer multiplications. In these, two operations such as depthwise convolution and pointwise convolution are performed sequentially.  Table 1 shows the calculation of parameters and multi-add (multiplication and addition) operations of the standard convolution operation and depthwise separable convolution.Table 2 shows the computation cost of standard convolution and depthwise separable convolution. Tables 1 and 2 show that computation cost is reduced by 8-9 times.

Here, DK = size of kernel = 3, DF = size of image characteristics, feature map = 14, *P* = total number of input channels = 512, and *Q* = total number of output channels = 512.

The above-declared values are used for the calculation of parameters and million multi-adds.

Figure 5 and Table 3 show the architecture of MobileNet V1 [30]. The first layer is the convolution layer with a stride value equal to two. Following that, the depthwise and pointwise layers take turns. The stride of the depthwise layer is one and two, respectively, to reduce the data's dimension (width and height) as it moves through the network model. The pointwise layer doubles the number of channels in the data. A ReLU activation function follows each of the convolutional layers. The said process repeats until the original image size 224 × 224 is reduced to 7 × 7 pixels with 1024 channels. Lastly, an average pooling operation has been performed that ends up with an image of dimension 1 × 1 × 1024. The following hyperparameters are used to reduce the network size and, in turn, make the network faster.

1. The width multiplier is denoted by *α*, where *α* between 0 and 1 is used to control the channel depth or a number of channels.
2. The resolution multiplier is denoted by *ρ*, where *ρ* between 0 and 1 is used to control an input image's dimension.

### 3.2. RPN

RPN (Figure 6) takes the input of any size and generates proposals created by sliding a small network over the output of the last layer of the image characteristic map. Its objective is to create a series of proposals, each of which is likely to have an object within it, and also define the class/label of the object, such as foreground or background. RPN uses nine bounding boxes to limit the image characteristic map, and all are multiplex of three to the reference bbox. Suppose the reference size of the box is 16 pixels, and the length and breadth are *l* and *w*, respectively. It then creates three anchor boxes with *l* : *w* ratios of 1 : 1, 1 : 2, and 2 : 1, as well as corresponding anchor boxes with dimensions of 8 pixels and 32 pixels. These anchor boxes are in charge of generating a series of bboxes of various sizes and aspect ratios referred to during object location predictions. These boxes are useful in detecting multiple objects, objects of different sizes, and overlapping objects. The bboxes are chosen based on the intersection over union (IOU) ratio between *P* and *Q*. Here *P* and *Q* indicate the bboxes and the ground-truth (GT) boxes. The formula for intersection over union is given below.

(5) $$\begin{array}{c} \text{IOU}=\frac{\text{area of overlap between }P\text{ and }Q}{\text{area of union of }P\text{ and }Q}. \end{array}$$

Then, NMS sorts these bounding boxes by their probability score and eliminates the boxes with IOU < 0.5.

RETRACTED

### 3.3. ROI Align

The proposals generated from RPN are of different sizes and aspect ratios; these need to be standardized to a fixed size to extract features. Faster R-CNN [60] uses the ROI pooling concept to generate fixed-size feature vectors from the feature map. ROI pooling works by dividing the ROI frame of dimension height *x* width into the *H* × *W* feature map of size height/*H* × width/*W*, and then the max-pooling operation is used in each subframe. Each channel of the feature map is pooled separately. In ROI pooling, to map the generated proposal to exact *x* and *y* index values, quantization operations such as floor and ceiling operations are performed to get the whole number for *x* and *y* index values. The ROI and extracted features are misaligned as a result of these quantizations. In order to remove the quantization problem, ROI align (Figure 7) was introduced in Mask R-CNN [61], which uses bilinear interpolation to calculate exact indexes for feature vectors. The proposal is divided into a predetermined number of smaller regions. In each region, four points are sampled; for each sampled point, the feature value is computed with bilinear interpolation.

## 4. Datasets

The proposed model or work is tested on various datasets shown in Table 4 which are COVERAGE [33], CASIA 1.0 [34], CASIA 2.0 [34], COLUMBIA [35], MICC F220 [36], MICC F600 [36], and MICC F2000 [36]. The COVERAGE [33] dataset includes 100 original-forged TIFF image pairs having resolution 400 × 486 where each original image contains SGOs (similar-but-genuine objects), making it difficult to differentiate between forged from genuine objects. This dataset is created by applying various postprocessing operations and a combination of these postprocessing operations to authenticate images. The postprocessing operations used for the creation of these forged images are scaling, translation, rotation, and addition of light effect addition. Ground-truth masks are available for this dataset. It also provides the degree of tampering or resemblance between the original and tampered images for all image pairs in the dataset. Sample images for this are shown in Figure 8.

RETRACTED

The CASIA dataset [34] comprises more tampering images; in this dataset, all the tampering images are color produced using Adobe Photoshop CS3 version 10.0.1 on Windows XP. This dataset has two versions, i.e., CASIA 1.0 and CASIA 2.0. The CASIA 1.0 dataset contains 1725 JPEG color images with a dimension of 384 × 256 pixels, and there are 800 genuine images and 925 tampered images in this dataset. Authentic images are roughly grouped into eight categories such as animal, architecture, scene, texture, plant, nature, and character. The tampered images are produced by applying splicing operations on authentic images by utilizing Adobe Photoshop.

CASIA 2.0 [34] is made up of 12614 images, in which some images are uncompressed TIFF and BMP, and others are JPEG with various *Q* factors of size in pixels ranging from 320 × 240 to 800 × 600. There are 7491 original images and 5123 tampered images in this dataset. Authentic images are roughly grouped into nine categories such as animal, architecture, scene, texture, plant, nature, character, and indoor. The tampered images contain both copy move and spliced images. However, these two datasets do not provide corresponding ground-truth masks, and for these two datasets, ground-truth masks are generated using VIA (VGG Image Annotator) [70], an open-source annotation tool that can specify regions in an image and generate textual information of those regions. Sample images for CASIA 1.0 and CASIA 2.0 are shown in Figures 9–11.

COLUMBIA [35] has 363 images; here, 183 are genuine images and 180 are spliced images. This dataset is created with four camera-captured images. Cameras used to create this dataset are Canon G3, Canon EOS 350D Rebel XT, Nikon D70, and Kodak DCS330. The images are all in JPG format, ranging in size from 757 × 568 to 1152 × 768 pixels; categories for these images are mainly desks, computers, or corridors.

MICC F220 [36] shows 220 images in this dataset, out of which 110 are original, and the rest 110 are forged. The image's size ranges from 722 × 480 to 800 × 600 pixels, with the forged region accounting for about 1.2% of the whole image area. Forged images in MICC F220 are created by randomly picking a rectangular portion from an image, copying it, then applying various attacks such as translation, scaling, and rotation, and then this portion is pasted on to image.

RETRACTED

Forged images in MICC F600 [36] are generated by applying more realistic and difficult postprocessing operations; it contains 600 images, out of which 440 are genuine, and 160 images are forged with image sizes ranging from 800 × 533 pixels to 3888 × 2592 pixels. MICC F2000 [36] contains 2000 images, out of which 1300 are authentic, and 700 are forged ones. Each image's size is 2048 × 1536 pixels, with the forged region accounting for about 1.12% of the whole image area. The sample image is shown in Figure 12.

Multiple Image Splicing Dataset [69] contains 618 authentic and 300 realistic multiple spliced images of size 384 × 256 that have been processed with rotation and scaling operations. It also includes images from various categories, including animal, architecture, art, scene, nature, plant, texture, character, and indoor scene. In this dataset, ground-truth masks are also provided which specify spliced instances for given multiple spliced images.

## 5. Dataset Annotation

One of the most significant areas in computer vision is annotation, involving methods for labeling an image with a class. There are a variety of tools for loading the images and marking the objects using per-instance segmentation. This makes accurate localization much easier with the help of bounding boxes and by generating masks. Annotation files are used to store this information. Annotation is divided into two types:

1. Image-level annotation-binary class indicating whether an object is present in the image or not.
2. Object-level annotation-bounding box and class label around an object instance in the image.

The COCO annotation format is automatically understood by advanced neural network libraries (like Facebook's Detectron2). Understanding of how the COCO annotation format is represented is necessary in order to modify the existing datasets and to create the custom ones. The dataset uses instance-level segmentation for similar pixels, and for different entities of a class, a unique label is given. The VGG Image Annotator [70] is a small and lightweight image and video annotation tool running entirely in the web browser to generate pixelwise annotations for JSON format images. The VGG Image Annotator [70] is used to draw bounding boxes or polygons around objects in the images and videos to form a computer vision model's supervision dataset. The annotation details for the bounding box are stored in JSON format. The structure of the file is given below:

1. Filename: contains the name of the image file.
2. Size: contains the size of the image in pixels.

## 6. Experimental Environment Configuration

This section specifies the experimental setup for the proposed model. Tables 5 and 6 show system specifications of the training environment. All experiments are conducted using Google Colab environment with specifications such as NVidia 1 × Tesla K80, compute capability 3.7, having 2496 CUDA cores with 12GB GDDR5 VRAM; the operating environment has 1 × single core hyper threaded Xeon Processors @2.3Ghz, i.e., (1 core, 2 threads) with 13 GB RAM. For performing experiments, Tensorflow 1.8.0, a deep learning framework, and Python 3.7 programming language are used. COCO pretrained network [71] is used for the generalization of parameters.  Table 7 shows a few configuration parameters which were modified from the original Mask R-CNN. In this experiment, a total of 3000 images are used for training, and 700 images are used for testing purposes. The training images are sized to retain their aspect ratio. The mask size is 28 × 28 pixels, and the size of the image is 512 × 512 pixels. This approach varies from the initial Mask R-CNN [39] approach, where image resize is done in such a way that 800 pixels are regarded as the smallest size and 512 pixels are trimmed to the highest. Bbox(bounding box) selection is made by considering IOU, which is the ratio of expected bboxes to ground-truth boxes (GT boxes). Mask loss considers only positive ROI and is an intersection of ROI and its ground-truth mask. Each mini-batch contains one image per GPU, with each image having an ROI of *N* samples and a 1 : 3 plus or minus ratio. The C4 backbone has a value of 64, while FPN has a value of 512. A batch size of one was maintained on a single GPU unit. The model was trained for 360 iterations with an initial learning rate of 0.01 and then modified to 0.003 at epoch 120 and 0.001 at epoch 240. Stochastic gradient descent (SGD) is used for optimization, with momentum initialized to 0.9 and weight decay initialized to 0.0001.

RETRACTED

## 7. Results

Various IOUs are used to measure the average precision (AP). Tables 8 and 9 show mean average precision for copy move and image splicing detection. In COCO, IoU values change from 50% to 95%, at a step of 5%. So it is end up with 10 precision-recall pairs. If we take the average of those 10 values, we get AP@[0.5:0.95]. The popular IOU scores are 50% (IOU = 0.5) and 75% (IOU = 0.75), interpreted as AP50 (AP_0.5_) and AP75 (AP_0.75_). *F*_1_-score (a pixel localization metric) is the evaluation metric criterion. Mask IOU is used to evaluate AP, and the *F*_1_-score is defined as follows:

(6) $$\begin{array}{c} F_{1}-\text{score}=\frac{2\times \left(\text{precision}*\text{recall}\right)}{2\times \left(\text{precision}+\text{recall}\right)}. \end{array}$$

Figures 13–15 show the ROC plots on COVERAGE [33], CASIA 1.0 [34], and CASIA 2.0 [34] datasets, respectively, for image forgery identification.

### 7.1. ROC AUC Curve

ROC AUC curves classify the given pixel as authentic or forged one. The proposed model classifies forged pixels with high confidence. The trade-off between the true positive rate (pixels correctly masked) and the false positive rate (pixels incorrectly masked) for our Mask R-CNN model using various probability thresholds is represented by ROC Curves. The graph shows false + rate (*x*-axis) vs. the true + rate (*y*-axis) for various candidate threshold values ranging from 0.0 to 1.0. It plots the rate of incorrectly segmented pixels to the rate of correctly segmented pixels. AUC is the area under the ROC curve. AUC with values [0.92, 1] [0.95, 0.1] have good effect, and AUC with [0.9, 1] has an average effect.

### 7.2. Precision-Recall Plots

Figures 16–18 show the precision-recall plots for the masks generated by the proposed technique on COVERAGE [33], CASIA 1.0 [34], and CASIA 2.0 [34] datasets. Different threshold values lead to changes in precision and recall. The high recall value indicates a larger area under the curve showing minimum FPR which shows improper masking of pixels, and minimal FNR means absence of mask pixels for which they should be present.

### 7.3. Comparison of Results with Mask R-CNN Using Various Datasets and Backbone Networks

As shown in Table 10, the overall number of parameters in the Mask R-CNN using ResNet-101 as a backbone network is substantially higher than that in the proposed technique.  Table 11 shows the training time and inference time comparison of ResNet-101 and MobileNet V1 on copy move and image splicing datasets. In terms of training time and inference time, Tables 11 and 12 indicate that MobileNet V1 outperforms ResNet-101. MobileNet V1 contains less trainable parameters and is computationally simpler in terms of parameter space usage, allowing it to make the most use of the existing parameters. As a result, MobileNet V1 outperforms in terms of training and inference times. In Tables 11 and 12, TT indicates training time in minutes and IT indicates inference time in milliseconds.

We evaluated the proposed Mask R-CNN model on various datasets and backbone network ResNet-101 for copy move and image splicing detection.  Table 13 shows a comparative analysis of Mask R-CNN with ResNet-101 and MobileNet V1 for precision, recall, and *F*_1_-score on standard datasets such as COVERAGE, CASIA 1.0, CASIA 2.0, MICC F220, MICC F600, MICC F2000, and COLUMBIA datasets. In terms of *F*_1_-score, the proposed model outperforms the ResNet-101 without the Sobel filter specified in the literature [39]. The *F*_1_-score of the proposed technique and the technique specified in the literature [39] is equal but the number of parameters of the proposed technique is less compared to the literature technique.

RETRACTED

Figures 19 and 20 show *F*_1_-score, precision, and recall for copy move and image splicing on various datasets using backbone networks such as ResNet-101 and MobileNet V1. The *x*-axis represents the model with *F*_1_-score, precision, and Recall, and the *y*-axis corresponds to evaluated metrics.

Table 14 shows a comparative analysis of AP, AP_0.5,_ and AP_0.75_ on standard datasets such as COVERAGE, CASIA 1.0, CASIA 2.0, MICC F220, MICC F600, MICC F2000, and COLUMBIA datasets using Mask R-CNN with ResNet-101 and MobileNet V1 as a backbone network. Here, for AP_0.5_, IOU = 0.5, and for AP_0.75_, IOU is = 0.75. Figures 21 and 22 show AP, AP_0.5,_ and AP_0.75_ for copy move and image splicing on various datasets using backbone networks ResNet-101 and MobileNet V1, where the *x*-axis represents the model with various average precision values and *y*-axis corresponds to evaluated metrics.  Table 12 shows that in terms of the average precision values, the proposed model on standard datasets considerably outperforms the existing architecture specified in literature [39] for identification and detection of copy move forgery. It also shows that in terms of average precision values, the proposed model outperforms the ResNet‐101 without the Sobel filter, specified in the literature [39]. In the case of identification and detection of image splicing forgery, average precision values of the proposed model and the existing model without the Sobel filter specified in the literature [39] are equal but the number of parameters of the proposed model is comparatively less.

Tables 8 and 9 show the mean average precision for copy move and image splicing detection on standard datasets. In the case of identification and detection of copy move forgery, precision values of the proposed model and the existing model without the Sobel filter specified in the literature [35] are equal but the number of parameters of the proposed model is comparatively less.

Figure 23 shows sample outputs of copy move, splicing forgery detection, and forged percentage of the image. The results show that the bounding box surrounds the object along with class (forged). It also gives a forged percentage of a region in an image and an accuracy percentage of copy move and splicing forgery detection.

## 8. Conclusion

This work presents a lightweight model, Mask R-CNN with MobileNet V1, for detecting and identifying copy move and image splicing [72] forgeries. We have used standard datasets such as COVERAGE, CASIA 2.0, MICC F220, MICC F600, MICC F2000, COLUMBIA, and CASIA 1.0 to evaluate the proposed model for copy move and image splicing forgeries. The proposed model outperforms ResNet-101 and achieves an *F*_1_-score of 70% on the MICC F600 dataset for copy move and 64% on CASIA 1.0 for image splicing. It also achieves average precision of 90% on MICC F2000 and COVERAGE for copy move and 90% for image splicing on the COLUMBIA dataset. The overall configuration was computationally more efficient than ResNet-101 [39]. According to experiments, the proposed approach effectively balanced efficiency and computational costs as compared to ResNet-101 [39]. It also provides the forged percentage of a region in an image. In the future, we are planning to extend this work for multiple image splicing and comparison of results with GAN-based architecture.

RETRACTED

## Figures and Tables

**Figure 1:** Digital image forgery detection.

**Figure 2:** Proposed architecture for detection and identification of copy move and image splicing forgery.

**Figure 3:** Standard convolution process.

**Figure 4:** Depthwise separable convolution [31, 32].

**Figure 5:** The architecture of MobileNet V1 [30].

**Figure 6:** Region proposal network.

**Figure 7:** ROI align.

**Figure 8:** Sample images from COVERAGE dataset [64]. (a) Light effect/illumination change. (b) Scaling operation ∅=0.8. (c) Rotation operation *θ*=10°.

**Figure 9:** Sample images from CASIA 1.0 dataset [65].

**Figure 10:** Sample images from CASIA 1.0 dataset [65].

**Figure 11:** Sample images from CASIA 2.0 dataset [65].

**Figure 12:** Sample image from MICC F2000 dataset [67]. (a) Original image. (b) Forged image without attack. (c) Forged image with scaling operation. (d) Forged image with the rotation operation.

**Figure 13:** ROC curve on COVERAGE dataset.

**Figure 14:** ROC plot on CASIA 1.0 dataset.

**Figure 15:** ROC plot on CASIA 2.0 dataset.

**Figure 16:** Precision-recall plot on COVERAGE dataset.

**Figure 17:** Precision-recall plot on CASIA 1.0 dataset.

**Figure 18:** Precision-recall plot on CASIA 2.0 dataset.

**Figure 19:** Comparison of *F*_1_-score, precision, and recall for copy move using backbone networks ResNet-101 and MobileNet V1.

**Figure 20:** Comparison of *F*_1_-score, precision, and recall for image splicing using backbone networks ResNet-101 and MobileNet V1.

**Figure 21:** Comparison of AP, AP0.5, and AP0.75 for copy move using backbone networks ResNet-101 and MobileNet V1.

**Figure 22:** Comparison of *F*_1_-score, precision, and recall for image splicing using backbone networks ResNet-101 and MobileNet V1.

**Figure 23:** Result of copy move and image splicing.

RETRACTED

**Table 1:** Calculation of parameters and million multi-adds [31, 32].

Standard convolution operation	Depthwise separable convolution
#Total params = (DK × DK × *P* + 1) × *Q* = (3 × 3 × 512 + 1) × 512 = 2.36*M* #Total multi-adds = (DF × DF) × #params = (14 × 14) × 2.36 *M* = 462*M*	Depthwise filters#Param = (DK × DK + 1) × *P* = (3 × 3 + 1) × 512 = 5120 #Multi-adds = (DF × DF) × #params = (14 × 14) × 5120 = 1*M*
	1 × 1 conv filters #Param = (1 × 1 × *P* + 1) × *Q* = (1 × 1 × 512 + 1) × 512 = 262656 #Multi-adds = (DF × DF) × #params = (14 × 14) × 262656 = 51.3*M* #Total params = 5120 + 262656 = 0.27*M* #Total multi-adds = 1*M* + 51.3*M* = 52.3*M*

**Table 2:** The computation cost of standard convolution and depthwise separable convolution.

Types of convolution	Million multi-adds	Million parameters
Standard convolution	462	2.36
Depthwise separable convolution	52.3	0.27

**Table 3:** MobileNet V1 architecture [30].

Type	Stride value	Filter shape	Input size
Standard convolution	Stride = 2	3 × 3 × 3 × 32	224 × 224 × 3
Depthwise separable convolution	Stride = 1	3 × 3 × 32	112 × 112 × 32
Standard convolution	Stride = 1	1 × 1 × 32 × 64	112 × 112 × 32
Depthwise separable convolution	Stride = 2	3 × 3 × 64	112 × 112 × 64
Standard convolution	Stride = 1	1 × 1 × 64 × 128	56 × 56 × 64
Depthwise separable convolution	Stride = 1	3 × 3 × 128	56 × 56 × 128
Standard convolution	Stride = 1	1 × 1 × 128 × 128	56 × 56 × 128
Depthwise separable convolution	Stride = 2	3 × 3 × 128	56 × 56 × 128
Standard convolution	Stride = 1	1 × 1 × 128 × 256	28 × 28 × 128
Depthwise separable convolution	Stride = 1	3 × 3 × 256	28 × 28 × 256
Standard convolution	Stride = 1	1 × 1 × 256 × 256	28 × 28 × 256
Depthwise separable convolution	Stride = 2	3 × 3 × 256	28 × 28 × 256
Standard convolution	Stride = 1	1 × 1 × 256 × 512 3 × 3 × 512	14 × 14 × 256
$5\times \begin{array}{c} \begin{array}{c} \text{depthwise separable convolution}\\ \text{convolution } \end{array} \end{array}$	Stride = 1	1 × 1 × 512 × 512	14 × 14 × 512 14 × 14 × 512
Depthwise separable convolution	Stride = 2	3 × 3 × 512	14 × 14 × 512
Standard convolution	Stride = 1	1 × 1 × 512 × 1024	7 × 7 × 512
Depthwise separable convolution	Stride = 2	3 × 3 × 1024	7 × 7 × 1024
Standard convolution	Stride = 1	1 × 1 × 1024 × 1024	7 × 7 × 1024
Average pool	Stride = 1	Pool 7 × 7	7 × 7 × 1024
Fully connected	Stride = 1	1024 × 1000	1 × 1 × 1024
Softmax activation function	Stride = 1	Classifier	1 × 1 × 1000

**Table 4:** Datasets used for experiment.

Name of datasets	Type of forgery	Total number of images	Size of image	Format of images
COVERAGE [33]	Copy move	100 (100 original-forged image pairs)	400 × 486	TIFF
CASIA V 1.0 [34]	Splicing	1725 (800 authentic images and 925 spliced images)	384 × 256 and 256 × 384	JPEG
COLUMBIA [35]	Splicing	363 (183 authentic images and 180 spliced images)	757 × 568 to 1152 × 768	BMP
CASIA V 2.0 [34]	Copy move, splicing	12614 (7491 authentic images and 5123 forged images)	320 × 240 to 800 × 600	BMP and TIFF uncompressed images. JPEG images with different *Q* factors.
MICC F220 [36]	Copy move	220 (110 original and 110 forged images)	374 × 256	JPEG
MICC F600 [36]	Copy move	600 (440 original and 160 forged images	800 × 533 to 3888 × 2592	JPEG
MICC F2000 [36]	Copy move	2000 (1300 original and 700 forged images)	2048 × 1536	JPEG
MISD [69]	Multiple image splicing	918 (618 original and 300 multiple spliced images	384 × 256	JPG

RETRACTED

**Table 5:** GPU specifications of the training environment.

Parameter	Specification
GPU	Nvidia K80/T4
GPU memory	12 GB
GPU memory clock	0.82 GHz/1.59 GHz
Performance	4.1 TFLOPS/8.1 TFLOPS
No. of CPU cores	2
RAM	12 GB

**Table 6:** CPU specifications of the training environment.

Parameter	Specification
CPU model name	Intel® Xeon®
CPU freq.	2.30 GHz
CPU family	Haswell
No. of CPU cores	2
RAM	12 GB

**Table 7:** Configuration parameters of the proposed model.

Parameters	Values
BACKBONE	mobilenetv1
IMAGE MAX DIM	512
IMAGE META SIZE	15
IMAGE MIN DIM	800
IMAGE SHAPE	[512, 512, 3]
LEARNING RATE	0.01
MASK SHAPE	[28, 28]
RPN_ANCHOR_SCALES	(8, 16, 32, 64, 128)
STEPS PER EPOCH	50
WEIGHT DECAY	0.0001

**Table 8:** AP comparison on five standard datasets using MASK R-CNN with MobileNet V1 as a backbone for copy move detection.

Method	Backbone	Avg. precision	COVERAGE	CASIA 2.0	MICC F220	MICC F600	MICC F2000	Mean
Mask R-CNN	ResNet-101	AP	0.60	0.60	0.90	0.70	0.90	0.76
	MobileNet V1	AP	0.90	0.60	0.90	0.70	0.90	0.80

**Table 9:** AP comparison on two standard datasets using MASK R-CNN with MobileNet V1 as a backbone for image splicing detection.

Method	Backbone	Avg. precision	COLUMBIA	CASIA 1.0	Mean
Mask R-CNN	ResNet-101	AP	0.70	0.90	0.80
	MobileNet V1	AP	0.90	0.70	0.80

**Table 10:** Comparison of ResNet-101 and MobileNet V1 in terms of parameters

Method	Backbone	Parameters	Trainable	Non-trainable
Mask R-CNN	ResNet-101	63,733,406	63,621,918	111,488
	MobileNet V1	**23,812,574**	**23,784,542**	**28,032**

**Table 11:** Training time and inference time comparison of ResNet-101 and MobileNet V1 on copy move datasets.

Model	Number of layers of model	Copy move datasets									
		COVERAGE		CASIA 2.0		MICC F220		MICC F600		MICC F2000	
		TT	IT	TT	IT	TT	IT	TT	IT	TT	IT
ResNet-101	347	432	610	508	656	505	620	515	612	665	628
MobileNet V1	**92**	**220**	**429**	**315**	**478**	**260**	**415**	**320**	**435**	**402**	**420**

**Table 12:** Training time and inference time comparison of ResNet-101 and MobileNet V1 on image splicing datasets.

Model	Number of layers of model	Image splicing			
		COLUMBIA color		CASIA 1.0	
		TT	IT	TT	IT
ResNet-101	347	504.40	660	520.78	684
MobileNet V1	**92**	**295.20**	**450**	**280.10**	**436**

RETRACTED

**Table 13:** *F*_1_-score, precision, and recall comparison analysis of Mask R-CNN with the backbone networks ResNet-101 and MobileNet V1 on various datasets for copy move and image splicing.

Type of forgery	Dataset	ResNet-101			MobileNet V1		
		*F*_1_-score	Precision	Recall	*F*_1_-score	Precision	Recall
Copy move	COVERAGE	0.54	0.59	0.60	0.61	0.60	0.63
	CASIA 2.0	0.64	0.76	0.62	0.68	0.70	0.66
	MICC F220	0.64	0.55	0.75	0.67	0.61	0.75
	MICC F600	0.70	0.72	0.65	0.70	0.75	0.68
	MICC F2000	0.66	0.50	0.77	0.64	0.54	0.80

Image splicing	CASIA 1.0	0.61	0.67	0.66	0.64	0.61	0.68
	COLUMBIA	0.63	0.65	0.62	0.61	0.60	0.63

**Table 14:** AP comparison analysis of Mask R-CNN with the backbone networks ResNet-101 and MobileNet V1 on various datasets for copy move and image splicing.

Type of forgery	Dataset	ResNet-101			MobileNet V1		
		Avg. precision	Avg. precision_0.5_ (AP_0.5_)	Avg. precision_0.75_ (AP_0.75_)	Avg. precision	Avg. precision_0.5_ (AP_0.5_)	Avg. precision_0.75_ (AP_0.75_)
Copy move	COVERAGE	0.60	0.65	0.58	0.90	0.92	0.80
	CASIA 2.0	0.66	0.74	0.75	0.60	0.65	0.80
	MICC F220	0.90	0.90	0.80	0.90	0.93	0.83
	MICC F600	0.78	0.80	0.74	0.70	0.74	0.60
	MICC F2000	0.90	0.90	0.72	0.90	0.90	0.76

Image splicing	CASIA 1.0	0.70	0.72	0.66	0.70	0.75	0.63
	COLUMBIA	0.90	0.95	0.79	0.90	0.92	0.77

## Data Availability

All the datasets used for experiments are publicly available. Links for the datasets are as follows: CASIA 1.0 and 2.0—https://www.kaggle.com/sophatvathana/casia-dataset; MICC datasets—https://lci.micc.unifi.it/labd/2015/01/copy-move-forgery-detection-and-localization/; COVERAGE—https://github.com/wenbihan/coverage; COLUMBIA—https://www.ee.columbia.edu/ln/dvmm/downloads/AuthSplicedDataSet/AuthSplicedDataSet.htm; and MISD—https://doi.org/10.5281/zenodo.5525829.

## Abbreviations

DL: Deep learning
CV: Computer vision
CNN: Convolutional neural network
FCN: Fully convolutional network
SVM: Support vector machine
RPN: Region proposal network
ROIs: Regions of interest
Mask R-CNN: Mask regional convolutional neural network
DSCLs: Depthwise separable convolution layers
bbox: Bounding box
NMS: Non-max suppression
IOU: Intersection over union.
